The article "Circular RNA NF1-419 enhances autophagy to ameliorate senile dementia by binding Dynamin-1 and Adaptor protein 2 B1 in AD-like mice" was retracted in 2025. Reasons: duplicated images; unreliable results or conclusions; concerns about the authorship.

# Circular RNA NF1-419 enhances autophagy to ameliorate senile dementia by binding Dynamin-1 and Adaptor protein 2 B1 in AD-like mice

**DOI:** 10.18632/aging.102529

**Published:** 2019-12-20

**Authors:** Chen Diling, Guo Yinrui, Qi Longkai, Tang Xiaocui, Liu Yadi, Yang Xin, Hu Guoyan, Shuai Ou, Yong Tianqiao, Wang Dongdong, Xie Yizhen, Burton B. Yang, Wu Qingping

**Affiliations:** 1 State Key Laboratory of Applied Microbiology Southern China, Guangdong Provincial Key Laboratory of Microbial Culture Collection and Application, Guangdong Open Laboratory of Applied Microbiology, Guangdong Institute of Microbiology, Guangdong Academy of Sciences, Guangzhou 510070, China; 2 Research and Development Institute of Chinese Materia Medica, Guangdong Pharmaceutical University, Guangzhou 510006, China; 3 Department of Pharmacy, The Fifth Affiliated Hospital of Guangzhou Medical University, Guangzhou 510700, China; 4 Sunnybrook Research Institute, Department of Laboratory Medicine and Pathobiology, University of Toronto, Toronto, Canada

**Keywords:** circular RNA, aging, astrocyte, biological function, autophagy

## Abstract

Recent studies have demonstrated circular RNAs (circRNAs) to be widely expressed and to have important physiological functions. However, the expression, regulation, and function of circRNAs in neuroglial cells are unknown. Herein, we characterized the expression, regulation, and function of circRNAs in astrocytes. Astrocyte circRNAs were identified by computational analysis of newborn SD rat primary astrocytes cultured with 20 g/L D-galactose. In this manner, 7376 circRNAs were identified, among which most circRNAs (5754) were derived from annot_exons, whereas 27 were antisense, 853 were exon/intron, 329 were intergenic, 41 were intronic, and 372 were one exon. Among these, *circNF1-419* was demonstrated to regulate autophagy, in over-expressing *circNF1-419* transfected astrocytes, through the PI3K-I/Akt-AMPK-mTOR and PI3K-I/Akt-mTOR signaling pathways. An adenovirus associated virus packaging system (virus titer 1 ×10^12^), over-expressing *circNF1-419* and injected into mouse cerebral cortex, showed autophagy enhancing activity by binding the proteins Dynamin-1 and Adaptor protein 2 B1 (AP2B1). This binding regulated aging markers (p21, p35/25, and p16) and inflammatory factors (TNF-α and NF-κB), and reduced the expression of Alzheimer’s disease marker proteins (Tau, p-Tau, Aβ_1-42_, and APOE), which delayed senile dementia. Transcriptome analysis of the brain showed that *circNF1-419* improved other signaling pathways, especially those related to the synapses of SAMP8 mice. These findings provide novel insights into *circNF1-419* and its potential usefulness for the diagnosis and treatment of dementia by regulating Dynamin-1 and AP2B1 mediated autophagy.

## INTRODUCTION

As the Chinese population ages, demographics will change such that by the end of 2020 the number of people over 60 years of age will be 19.3 percent and by 2050 greater than 38 percent of the total population. Retirement presents numerous serious problems, which will require intensive investigation into not only age-related disease, but also strategies and measures to serve the elderly.

Aging is a subclinical pathogenesis, which is an interplay between multiple invariant genes and variable environments. Symptoms develop slowly and include; cognitive decline, brain aging, and visceral degenerative diseases. Aging is closely linked to diseases of aging including; hypertension, stroke, diabetes, cancer, and neurodegenerative diseases such as Parkinson's disease and dementia, which are common risk factors for age-related disease [1–5]. Understanding the dynamic changes during the aging of the brain at the cellular and molecular level is one of the most complicated and profound subjects in contemporary life science. The involvement of neurogliocytes in the process of brain aging has been noted [6, 7], although their relationship to ageing and disease is not well established.

Glial cells are widely distributed in the central nervous system, accounting for approximately half of brain weight, if neurons are excluded. Glial cells participate in almost all nervous system activities from the embryonic stage to the aged brain. They are involved in central nervous system functions including; synaptic transmission, nerve tissue repair, regeneration, immunity, and aging. Glial cells are associated with various neurological diseases and are equal functional partners with neurons [8–13]. Glial cells form the microenvironment of the central nervous system and are activated with aging. Microglia can secrete the protein Tau via exosomes both *in vitro* and *in vivo*. Inhibition of exosome secretion can significantly reduce the diffusion of Tau. Exosomes secreted by these cells contain miRNA, circRNA, and other secretory products that influence physiological function [14, 15]. Further, clearance of senescent glial cells can prevent tau-dependent pathology and cognitive decline [16]. These results suggest that targeting senescent cells could provide a therapeutic avenue for the treatment of Alzheimer’s disease (AD).

Recent evidence suggests that circular RNA (circRNA) may be important for brain function in that CDR1 is found at high levels in mammalian neurons [17]. Further, circRNA transcripts produced by neurons accumulate in aging *Drosophila*. Increased levels of many circRNAs are observed when synapses form [18], which suggest that circRNAs may regulate synapse formation, and may be dynamic for life activities [19]. As a biomarker or drug target circRNA may be effective for treatment of neurodegenerative diseases, with evidence that CDR1 is reduced in AD [17]. For brain circRNAs there were are many questions that need to be answered regarding function including their effect on: gene expression, neuroplasticity, neurogenesis, and behavior. Herein, we devised a D-galactose glial cell aging model. This model was used to identify and characterize senescence-regulated astroglial circRNAs by bioinformatics, high-throughput sequencing, and polymerase chain reaction. Further, a targeted circRNA over-expression system was used to assess physiological function and the targeted effects of circRNA on the aging process. In this manner, new targets were assessed for the diagnosis and treatment of age-related brain disease.

## RESULTS

### Senescent astrocyte establishment and identification

To assess senescence-regulated circRNAs, a senescent cell aging model was required with the following characteristics. First, cells must die only from aging. Second, results must be repeatable. Senescent cells were prepared by continuous passage in culture with D-galactose at different concentration (0, 5, 10, 20, and 30 g/L). Senescence-associated β-galactosidase staining (procedure based on the kit’s instructions, Figure 1A–1D) and single cell gel electrophoresis were used to identify senescent cells [20–22] (Figure 1E, 1F). Cell morphology, by light microscopy, of Giemsa stained cells (Figure 1G) identified large amounts of cavitation and swelling. In a dose dependent manner, D-galactose inhibited cell growth (Figure 1H–1M). Based on previous reports, culture in 20 g/L D-galactose for two generations was chosen as the ideal culture conditions. Even through 20 g/L D-galactose for two generations decreased cellular proliferation, the number of available cells that stained positive met experimental demands (Figure 1G–1J). Cell cycle results are shown in Figure 1N. Expression of aging biomarkers, P21^Cip1/Waf1^ and P16^INK4a^, were increased (Figure 1O). These results demonstrate D-galactose to induce the senescence of astrocytes after two generations of cell culture (Figure 1A–1O).

**Figure 1:** **Senescent astrocyte establishment and identification.** (**A**–**D**) The astrocyte were treated with 20 g/L of D-galactose for different continuous passage culture time, and the senescent cells rate (bule staining cells) was detected using β-galactosidase staining; (**E**, **F**) The cells were treated with 20g/L of D-galactose for continuous passage culture of two generations, and the damaged DNA fragments was detected by single cell gel electrophoresis; (**H**–**K**) TUNEL (Terminal-deoxynucleoitidyl Transferase Mediated Nick End Labeling) staining and DAPI (4',6-Diamidino-2-Phenylindole, Dihydrochloride) staining, DAPI stained all cells blue and TUNEL kits labeled apoptotic cells with green fluorescence; (**L**) The cell proliferation rate, (**M**) apoptosis rate and (**N**) cell cycle measurement after treated with 20 g/L of D-galactose for different continuous passage culture time; (**O**) Western blotting of P16^INK4a^ and P21^Cip1/Waf1^ protein expressions; (**P**) The cell morphology with Giemsa staining at different time on the 20 g/L of D-galactose concentration. D0 (culture without 20 g/L D-galactose), D1 (culture in 20 g/L D-galactose for one generations) and D2 (culture in 20 g/L D-galactose for two generations) (Figure 2C, 2D), D3 (culture in 20 g/L D-galactose for three generations). Data are presented as the means±SD of 3 independent experiments. *p <0.05 and **p <0.01 *vs*. the control (normal or D0) group by one-way ANOVA, followed by the Holm-Sidak test.

### Senescence-regulated astroglial circRNAs

Astroglia circRNAs were identified in astroglia cells of newborn rats by consulting PYTHON scripts provided by circBase. There were 7376 circRNAs identified in this study. Most circRNAs (5754) were derived from annot_exons, 27 were antisense, 853 exon/intron, 329 intergenic, 41 intronic, and 372 exon (Figure 2A).

**Figure 2:** **CircRNAs expression in D-galactose-induced deficits astrocyte.** (**A**) 7376 astroglia circRNAs were identified and their types were showed; (**B**) Different expression of circRNAs in D-galactose induced aging astrocyte; (**C**) Time series analysis of circRNAs positively correlated to the degree of aging; Different expression of circRNAs in D2 (**D**); Aging regulates circRNAs as circ_NF1-419 (circ_000978), circ_002671, circ_003172, circ_CTGF-212, circ_SIRT1-395, circ_002276, circ_SIRT1-623, circ_001215, circ_001216 and circ_000987 were validated by reverse transcription polymerase chain reaction in cultured astrocyte (**E**, **F**). D0 (culture without 20 g/L D-galactose), D1 (culture in 20 g/L D-galactose for one generations) and D2 (culture in 20 g/L D-galactose for two generations) (Figure 2C, 2D), D3 (culture in 20 g/L D-galactose for three generations). Data are presented as the means ± SD of 3 independent experiments. **p <0.01 *vs*. the control group (D0) by one-way ANOVA, followed by the Holm-Sidak test.

Differentially expressed circRNAs in D-galactose induced aging astrocytes are shown in Figure 2B (*p* < 0.05 with greater than 2-fold change). These results demonstrate differential expressions of circRNAs in astrocytes with different degrees of aging. Compared to D0 (culture without 20 g/L D-galactose), 123 circRNAs were up-regulated in D1 (culture in 20 g/L D-galactose for one generations) and D2 (culture in 20 g/L D-galactose for two generations) (Figure 2C, 2D), which demonstrated these circRNAs to be positively related to the degree of aging. Some circRNAs were down-regulated at D3 (culture in 20 g/L D-galactose for three generations). Based on cell morphology (Figure 1D and Figure 1L–1N), we can conclude that cells at D3 were apoptotic or dead. These results confirm D-galactose induced senescence in astrocytes, treated for no less than two generations.

To assess the effects of circRNAs on aging, we chose D2 and D0 for analysis. CircRNAs with altered expression, *p* < 0.05 and greater than 1.5 folds change, were considered differentially expressed. There were 319 up-regulated (Figure 2D) and 643 down-regulated circRNAs (Supplementary Table 1) at D2.

D-galactose-induced circRNAs were validated by qRT-PCR (PCR primers in Supplementary Table 2) of cultured astrocyte including; *circ_NF1-419*, *circ_000987*, *circ_001215*, *circ_00121*, *circ_002276*, *circ_002671*, *circ_003172*, *circ_CTGF-212*, *circ_SIRT1-395,* and *circ_SIRT1-623.* All were increased by aging (Figure 2E), suggesting that these circRNAs accelerate the ageing process. We focused on the candidates that had the greatest differential expression between the cancerous and normal groups and matched them with circRNADb (Supplementary Table 1). Among these specific candidates, novel_circ*NF1-419* (mmu_circ_0003411), which was formed by circularization of chr17: 29483000-29490394 strand: + of the NF1 gene (RPKM 5.97 in D2, while 0 in D0), attracted our attention.

### CircNF1-419 enhances autophagy in astrocytes

To validate the essential role of *circ-NF1-419* in cell cycle, apoptosis, and cell proliferation, an over-expressing *circNF1-419*-transfected rat astrocyte was designed as described [23]. An 83bp framework sequence and an AG receptor were added upstream of the 419bp sequence of rno_circ_000978 (Supplementary Figure 4A, 4B). A GT donor and a 57bp frame sequence were added downstream, connecting the full-length sequence 575bps (Supplementary Figure 4Aa) to the pCDH-CMV-MCS-EF1-GFP+Puro (CD513B-1) vector (Supplementary Figure 4A, 4C) by XbaI and BamHI (Supplementary Figure 4A–4C). The sequence is shown in (Supplementary Figure 4A, 4D). A lentivirus packaging protocol was performed and an over-expressing *circNF1-419*-transfected rat astrocyte was finalized (Supplementary Figure 4B). As shown in Figure 3 *circNF1-419* influences on astrocyte proliferation (Figure 3A), apoptosis (Figure 3B), or cell cycle (Figure 3C). Western blot analysis (Figure 3D) showed the levels of Atg12, LC3A, LC3B in over-expressing *circNF1-419*-transfected rat astrocytes to be significantly different from wild type astrocytes, indicating that *circNF1-419* primarily influences autophagy. For confirmation, transmission electron microscopy demonstrated phagophore, endosome, autophagosome, amphisome, autolysosome, and lysosome formation in the over-expressing *circNF1-419*-transfected astrocytes, which were not observed in the vector control (Figure 3E).

**Figure 3:** **Essential roles of circ-NF1-419 on proliferation, apoptosis, cell cycle and autophagy test.** Influence on astrocyte proliferation (**A**), apoptosis (**B**), and cell cycle (**C**); Western blot analysis (**D**) showed the levels of Atg12, LC3A, LC3B in over-expressing *circNF1-419*-transfected rat astrocytes; (**E**) Transmission electron microscopic imaging showing autolysosomes (arrows) and autophagosomes with double-membraned autophagic vacuoles (arrowheads) in over-expression circNF1-419-transfected rat astrocyte. Scale bar: 5μm and 2μm. Data are presented as the means±SD of 3 independent experiments. **p <0.01 *vs*. the model group by one-way ANOVA, followed by the Holm-Sidak test.

### CircNF1-419 participates in the regulation of astrocyte autophagy

To identify the regulator of *circNF1-419* in autophagy, we identified key proteins involved in the autophagy signaling pathway by western blot. As shown in Figure 4 for over-expressing *circNF1-419*-transfected astrocytes, the level of mTOR was inhibited, levels of PI3Kp85, PI3Kp100, and AMPK were increased, p53 was slightly increased, while Erk1/2 did not change. Signal transduction pathway expressed proteins Atg13, ULK1, Beclin-1, Atg14, Atg5, Atg12, LC3A, LC3B I, and LC3B II were identified. The results show the PI3K/Akt pathway to converge on mTOR as a central regulator of Nf1 (gene-symbol for *circNF1-419*) [24]. Taken together these data suggest *circNF1-419* to regulate autophagy through PI3K-I/Akt-AMPK-mTOR and PI3K-I/Akt-mTOR signaling pathways, or possibly through factors upstream of these pathways. Precise targets and pathways will require additional study.

**Figure 4:** **CircNF1-419 participates in the regulation of autophagy in astrocyte.** The expression of PI3Kp85, PI3Kp100, AMPK, Atg13, ULK1, Beclin-1, Atg14, Atg5, Atg12, LC3A, LC3B I and LC3B II proteins in the over-expressing *circNF1-419*-transfected rat astrocyte were measured by using western blotting. Data are presented as the means±SD of 3 independent experiments. **p <0.01 *vs*. the WT by one-way ANOVA, followed by the Holm-Sidak test.

### CircNF1-419 delays senile dementia by enhancing autophagy in vivo

The function of *circNF1-419* was assessed *in vivo* after consideration of autophagy levels in age-related disease animal models. Then global brain tissue was dissected from 28-week-old SAMP8 and APP/PS1 mice (purchased from the Beijing HFK Bioscience Co., LTD [Certificate No: SCXK (Jing) 2014-0004]). Levels of Atg12, LC3A, LC3B I, and LC3B II proteins were detected by western blot [25]. As shown in Figure 5 the levels of Atg12, LC3A, LC3B I, and LC3B II protein in APP/PS1 and SAMP8 mice were lower than levels in normal C57 mice (*p* < 0.05), suggesting that the global brain autophagy levels of AD mice were disordered. Further, *Ganoderma lucidum* extracts (low dose group is LL; high dose group is LH) and *Hericium erinaceus* extracts (low dose group is HL; high dose group is HH) treated animals had enhanced autophagy levels. Alternatively, activation of autophagy may delay or prevent age-related diseases such as AD.

**Figure 5:** **Autophagy level in the age-related disease model animals.** The expression of Atg12 (**A**, **B**), LC3A (**A**, **C**), LC3B I (**A**, **D**) and LC3B II (**A**, **E**) protein in the 8 months old APP/PS1 and SAMP8 mice were measured using western blot (**A**–**E**). Data are presented as the means ± SD of 3 independent experiments. ^#^*p* <0.05 *vs*. the control group, **p <0.01 *vs*. the model group by one-way ANOVA, followed by the Holm-Sidak test.

Next, we designed an AAV viral transduction system with RNA interference (si*circNF1-419*-AAV, Supplementary Figure 5A, 5B) and separately an over-expressing *circNF1-419* (ss*circNF1-419*-AAV, Supplementary Figure 5C, 5D). Two μl of the AAV packaging system (virus titer 1 × 10^12^) were injected into the cerebral cortex of mice (SAMP8 mice, two week old new born KunMing mice, and 12 month old Balb/c mice). As expected, autophagy levels were significantly increased (LC3A, LC3B I, and LC3B II) for *circNF1-419*-OV-AAV injected mouse brains in comparison to control brains (*p* < 0.05, Figure 6A, Supplementary Figure 6, and Figure 7H). The si*circNF1-419*-AAV injected animals were slightly inhibited (Figure 6A), while AD marker proteins such as Tau, p-Tau, Aβ A4, APOE, and BACE1 were inhibited (*p* < 0.05, Figure 6B and Supplementary Figure 6), and the senescence-associated biomarkers p21 and p35 were improved (*p* < 0.05, Figure 6B and Figure 6) after treatment with *circNF1-419-OV-AAV* for 2 months. Neuropathological changes were also improved (Figure 6C), with some inflammatory factors, NF-κB and TNF-α, improved as judged by immunohistochemistry (Supplementary Figure 6, *p* < 0.05). The si*circNF1-419*-AAV showed no improvement and a worsening condition (Figure 6 and Supplementary Figure 6). These results and those derived from astrocytes suggest that *circNF1-419* can enhance autophagy levels and possibly improve AD related regulators.

**Figure 6:** **CircNF1-419 delays senile dementia by enhancing autophagy in vivo.** *CircNF1-419* up-regulates the autophagy biomarkers including LC3A I, LC3A II, LC3B I and LC3B II (**A**), and improves the AD related regulators including p-Tau, p-Tau (202), p-Tau (396), Aβ A4, APOE, BACE1, TNF-α, NF-κB and p21 (**B**); histopathological (**C**) examination of hippocampus (Ca-b) and cortex (Cc-d); and immunostaining examination (**D**) of LC3A in hippocampus (De) and cortex (Df). All densitometric data of proteins expression using ImageJ are presented as the means±SD of 3 independent experiments. **p <0.01 *vs*. the model group by one-way ANOVA, followed by the Holm-Sidak test.

**Figure 7:** ***CircNF1-419* enhances autophagy by binding dynamin-1 and AP2B1 protein in vivo.** *circNF1-419* can pull-down dynamin-1 and AP2B1 protein (**A**, **B**), the proteins of dynamin-1 and AP2B1 quantified using Wes™ and the Simple Western from ProteinSimple; and RNA binding protein immunoprecipitation assay showed that the dynamin-1 and AP2B1 protein can pull down the circNF1-419 (**C**, **D**); the computer-aided molecular simulation demonstrated that the dynamin-1 and AP2B1 protein binds the *circNF1-419* (**E**); the expression of dynamin-1 and AP2B1 protein in the whole brain tissues (**F**); *CircNF1-419* improves the brain transcriptome in AD mice (**G**); *CircNF1-419* levels in AAV viral transduction system with RNA interference and separately an over-expressing *circNF1-419* (**H**). Data are presented as the means±SD of 3 independent experiments. **p < 0.01 *vs*. the model group by one-way ANOVA, followed by the Holm-Sidak test.

### CircNF1-419 enhances autophagy by binding Dynamin-1 and Adaptor protein 2 B1 (AP2B1) proteins in vivo

To assess the precise targets and pathways by which *circNF1-419* regulates autophagy, fluorescent *in situ* hybridization (FISH) was used to detect [26] *circNF1-419*-*OV-AAV* in infected brain tissue (Supplementary Figure 7A and 7B). Results showed that *circNF1-419* was located in the cytoplasm, indicating that *circNF1-419* may bind proteins related to autophagy control. RNA pull down experiments were implemented using biotin-coupled *circNF1-419*. As shown in Figure 7A, binding-proteins were pulled down and identified by LC-MS (Supplementary Table 3). Western blot verified that Dynamin-1 and AP2B1 (two of five tested antibodies) proteins were found (Figure 7B) in both SAMP8 mice and KM mice. RIP using antibody against Dynamin-1 and AP2B1 showed that *circNF1-419* was pulled down (Figure 7C, 7D). By qRT-PCR, results were in agreement with computer-aided molecular simulation as showed in Figure 7E and with more detail, Supplementary Figure 8. Western blot analysis of whole brain tissue demonstrated Dynamin-1 and AP2B1 levels to be influenced by *circNF1-419* (Figure 7F, 7H). These results indicate that *circNF1-419* binds Dynamin-1 and AP2B1, and may influence the splicing of mRNA, polyadenylation, stabilization, localization, and translation (Figure 8). In sum, *circNF1-419* binds two proteins, influencing signal transduction and function.

**Figure 8:** **Role of circNF1-419 in regulated astrocyte and delay dementia.** Circular RNA NF1-419 has autophagy enhancing activity by binding Dynamin-1 and AP2B1, delaying senile dementia by regulating aging markers (p21, p35/25, p16) and inflammatory factors (IL-6, IL-10, NF-κB), and by reducing the expression of AD marker proteins Tau, p-Tau, Aβ_1-42_, BACE1 and APOE.

### CircNF1-419 improves the brain transcriptome of AD mice

To assess downstream regulatory molecules and/or signaling pathways, RNA-sequencing was performed. The RNA-sequencing analysis of SAMP8 mice showed that *circNF1-419*-*OV-AAV*: up-regulated *CHRM*, *ADR*, *DRD*, *HTR*, *AGTR*, *FPRL*, *CCKR* (Figure 7G and Supplementary Table 4); down-regulated *PTGDR*, *CNR1*, *GCGR*, *VIPR*, *GRM*, *GRIN*, *GRI* (Figure 7G and Supplementary Table 4); bi-directionally regulated GABR that influences neuroactive ligand-receptor interaction; and regulated others genes (Figure 7G and Supplementary Table 4) that influence other pathways including retrograde endocannabinoid signaling, glutamatergic synapse, calcium signaling pathway, cholinergic synapse, serotonergic synapse, GABAergic synapse, dopaminergic synapse, nitrogen metabolism, estrogen signaling pathway, circadian entrainment, long-term depression, inflammatory mediator regulation of TRP channels, long-term potentiation, and the PI3K-Akt signaling pathway (Supplementary Figure 9A, 9B, and Supplementary Table 4). All of these can be related to neurodegenerative diseases. These results suggest that *circNF1-419* binds Dynamin-1 and AP2B1, influencing multiple signaling pathways especial at the synapse. However further investigation is necessary to define mechanisms of regulation.

## DISCUSSIONS

Accumulating evidence supports a direct role for autophagy in the aging process, with multiple genetic experiments demonstrating the influence of autophagy-related genes on longevity [27–30]. Macroautophagy/autophagy failure, with the accumulation of autophagosomes, is an early neuropathological feature of AD that directly affects amyloid beta (Aβ) metabolism [31]. Dysfunction of presenilin 1 impairs lysosomal function and prevents autophagy flux. In this study, we also found that autophagy levels in the brain of 28 weeks old SAMP8 and APP/PS1 mice were abnormal (Figure 5). Previous studies suggested that enhancing autophagy may be a promising new therapeutic strategy for AD [32–34]. Although the etiology and pathogenesis of AD have not been elucidated completely, one of the most characteristic neuropathological changes is the formation of neurofibrillary tangles within senile plaques deposited by β amyloid protein with Tau hyper-phosphorylation within nerve cells, as well as neuronal loss accompanied by neuroglial hyperplasia [35]. Normally, glial cells support and protect neurons and participate in all neural activities, including central nervous system development, synaptic transmission, neural tissue repair and regeneration, neural tissues aging, neural immunity, and a variety of neurological diseases [36–38]. However, in the case of brain injury and/or disease, pathological changes and neuron death are often irreversible. In contrast, glial cells that are capable of division, could quickly respond to nerve damage, divide and form a layer or barrier in the lesion area, preventing the expansion of nerve injury. By this scenario, unfortunately, the central neurons would die and be replaced by glial cells that formed the glial scar, with loss of function. This is a serious problem that urgently needs to be solved [37–39]. Glial cells and neurons should be considered equally important partners within the brain [40]. Further, glial cells can prevent Tau-dependent pathology and cognitive decline [16], suggesting that enhanced glial cell autophagy could be an effective therapeutic strategy for AD.

In this study, we chose to assess circRNA targets in senescent glial cells in order to develop an effective therapeutic strategy for AD. First, a senescent astrocyte model using 20 g/L D-galactose in continuous passage culture was developed (Figure 1). RNA sequencing demonstrated 319 up-regulated and 643 down-regulated circRNA in this model, among which some circRNAs were increased with aging, suggesting that circRNAs could be biomarkers of aging. Next, we chose to assess *circNF1-419* for its function and influence on aging. Over-expression of *circNF1-419* in astrocytes (Figures 3 and 4), and the over-expression of the *circNF1-419* AAV system in 8 months old SAMP8 mice and 12 months old Balb/c mice (Figure 5) indicated that *circNF1-419* could enhance autophagy levels. AD marker proteins Tau, p-Tau, Aβ_1-42,_ and APOE were inhibited (Figure 6). Aging related regulators p21, p35/25, and p16 were changed. Inflammatory regulators TNF-α and NF-κB were changed. The si*circNF1-419*-AAV showed no improvement. These results indicate that *circNF1-419* may delay the progress of AD and defer senility, suggesting that enhanced autophagy could be an effective therapeutic strategy for AD.

Previous studies demonstrated that circRNAs can function as miRNA sponges that reduce levels of the targeted miRNAs [41]. Studies also revealed that circRNAs could bind, store, sort, and sequester proteins to particular subcellular locations, acting as dynamic scaffolding molecules that modulate protein-protein interactions [42], and coding for proteins [43]. In this study, we found no sponge miRNA nor coding protein functions of *circNF1-419* (chr17: 29483000- 29490394 strand: +). FISH showed that *circNF1-419* localized to the cytoplasm, suggesting a protein binding function. The RNA pull down experiments showed that *circNF1-419* could bind Dynamin-1 and AP2B1 protein in SAMP8 mice. The RIP experiments confirmed this binding function. In this study, AAV treated KM mice provided more evidences that *circNF1-419* could bind Dynamin-1 and AP2B1 proteins. Further, the in silico experiments demonstrated that *circNF1-419* could also bind Dynamin-1 and AP2B1 proteins. Previously, neurofibromin 1 (NF1) was shown to be a direct effector of GPCR signaling via Gβγ subunits in the striatum, regulating Ras pathways [44]. Dynamin-1 is a 100-kDa GTPase and *circNF1-419* could be a direct effector of Dynamin-1. Alternatively *circNF1-419* could bind Dynamin-1 and influence its function. Dynamin-1 can also be activated by Akt/GSK3β signaling, which was demonstrated in H1299 non-small lung cancer cells [45]. Dynamin-1 is an essential component of vesicle formation in receptor-mediated endocytosis, synaptic vesicle recycling, caveolae internalization, and vesicle trafficking in and out of the Golgi [46]. Studies also revealed that vesicles coated with clathrin and AP2B1 play an important role in internalization of receptors and their bound ligands during clathrin-dependent endocytosis and the fission of clathrin-coated vesicles (CCVs) from the plasma membrane, which are mediated by dynamin proteins. Dynamin-1 is also thought to provide a source of membranes for autophagosomes by pinching off vesicles from the plasma membrane (Ravikumar et al., 2010). Moreover, Dynamin-1 is required for the regeneration of lysosomes by pinching off membrane from autolysosomes in hepatocytes (Schulze et al., 2013). Dynamin-1 has also been proposed to complete the maturation of autophagosomes, leading to impairment in autophagy in Dynamin-1 mutant mice (Durieux et al., 2012). Hence, *circNF1-419* is a direct effector of Dynamin-1 and AP2B1 binding, which is followed by Dynamin-1 and AP2B1 protein mediated autophagy. Autophagy then regulates aging and inflammatory reactions, influencing the downstream expression of AD marker proteins Tau, p-Tau, Aβ_1-42_, APOE, and BACE1. These *in vitro* results indicate that *circNF1-419* could delay the progress of AD and defer senility by binding Dynamin-1 and AP2B1 and delaying autophagy.

In a four-vessel transient cerebral-ischemia rat model, memory impairment was associated with a decrease in expression of hippocampal Dynamin 1 [47]. In older people with cerebrovascular disease [48] Dynamin-1 was associated with both preserved cognition and regenerative responses. Dynamin-1 pharmacologic inhibition; impairs hippocampal-dependent associative memory, accentuates synaptic fatigue, reduces long- term potentiation, as well as post-tetanic potentiation, and neurotransmitter release [49]. Hence, Dynamin-1 as a key protein for modulation of memory. Studies also showed that Dynamin-1 could affect amyloid generation through regulation of BACE-1 subcellular localization and its enzymatic activity [50]. Further, soluble oligomeric Aβ, but not fibrillar Aβ, was responsible for sustained calcium influx, calpain activation, Dynamin-1 degradation [51], BACE-1 and Aβ modified expression (Figure 6).

This study identified 7376 circRNAs, among which most circRNAs (5754) were derived from annot_exons, whereas 27 were antisense, 853 exon/intron, 329 intergenic, 41 intronic, and 372 of one exon. Further, *circNF1-419* was shown to regulate autophagy in over-expressing *circNF1-419* transfected astrocytes, likely through PI3K-I/Akt-AMPK-mTOR and PI3K-I/Akt-mTOR signaling pathways. An AAV packaging system (virus titer 1 ×1 0^12^) over-expressing *circNF1-419,* when injected into mouse cerebral cortex, showed autophagy enhancing activity by binding Dynamin-1 and AP2B1, delaying senile dementia by regulating aging markers (p21, p35/25, p16) and inflammatory factors (IL-6, IL-10, NF-κB), and by reducing the expression of AD marker proteins Tau, p-Tau, Aβ_1-42_, and APOE in SAMP8 mice. Transcriptomic analysis of brains showed *circNF1-419* to improve other signaling pathways especial at the synapse in SAMP8 mice (Figure 8). These findings provide novel insights into the role of *circNF1-419* in dementia. These insights may be useful for diagnosis and treatment of disease.

## MATERIALS AND METHODS

### Senescent astrocyte preparation

Murine cerebral cortical cells from a 1-day-old rat were dissociated after a 30 min trypsinization (0.15%) in D-Hanks. The cells were centrifuged, washed, and plated in 75 cm^2^ culture flasks (1.5 × 10^5^/cm^2^) in Dulbecco's Modified Eagle *Medium (*DMEM)/F12 containing 12% fetal bovine serum (FBS), penicillin (100 U/ml), streptomycin (100 μg/ml), and B27 (Cyagen Biosciences, Suzhou, Jiangsu, China). The medium was replenished every 2 to 3 days after plating. On day 7 of culture, floating microglial cells and oligodendrocytes were removed after shaking at 280 rpm and 37°C for 18 h. Astroglia cells were harvested after trypsinization (0.15 % trypsin in Hank’s Balanced Salt Solution, HBSS) for 30 min. After adding FBS (final concentration 12%), centrifugation, and washing, the cells were seeded into new flasks with DMEM/F12 followed by a medium change after 24 h. This subculture procedure was repeated weekly 2 - 3 times to remove residual oligodendrocytes and microglia in order to achieve a highly purified astrocyte culture. The cells were plated into 48-well cell culture plates (1 × 10^5^ cells/well), under normal or 20 g/L D-galactose conditions.

### Animals

Male SAMP8 mice (5 months old, mean body weight 20 ± 5 g) were purchased from Beijing HFK Bioscience Co., LTD (Certificate No: SCXK [Jing] 2014-0004). All animals were allowed to acclimate for at least 1 week prior to the initiation of the experiments. Mice were randomly allocated into 3 groups of 8 animals each: SAMP8 model group, ss*circNF1-419*-OV-AAV infected group, and sh*circNF1-419*-OV-AAV infected group. Newborn KM mice and Balb/c mice were obtained from the Center of Laboratory Animals of Guangdong Province of China, (SCXK [Yue] 2008-0020, SYXK [Yue] 2008-0085) and pair-housed in plastic cages in a temperature-controlled (25 ± 2°C) colony room with a 12/12-h light/dark cycle. The animals had free access to food and water. All experimental protocols were approved by the Center of Laboratory Animals of the Guangdong Institute of Microbiology. All efforts were made to minimize the number of animals used.

### RNA isolation and sequencing

Total RNA was isolated using Qiazol and miRNeasy Kits, including additional DNase I digestion. Ribosomal RNA was removed using Ribo-Zero^TM^ Magnetic Gold Kit, with enzymatic degradation of linear RNA by RNase R enzyme. The first chain of cDNA was synthesized with six base random hexamers, with dNTPs, RNase H, and DNA polymerase I used to synthesize the second chain of cDNA. Purification was accomplished with a QiaQuick PCR kit, followed by elution with EB buffer after terminal repair, base A processing, and sequence joining. For next generation sequencing, 0.5 μg of ribosomal RNA-depleted RNA was fragmented and primed. Sequencing libraries were constructed using Illumina TruSeq RNA Sample Preparation Kits and were sequenced with an Illumina HiSeq^TM^ 2500 flowcell.

### Computational analysis of circRNAs

The reads were first mapped to the latest UCSC transcript set using Bowtie2 version 2.1.0 [52] and the gene expression level was estimated using RSEM v1.2.15 [53]. For lincRNA expression analysis, we used the transcripts set form Lncipedia (http://www.lncipedia.org). TMM (trimmed mean of M-values) was used to normalize gene expression. Differentially expressed genes were identified using the edgeR program [54]. Genes showing altered expression with *p* < 0.05 and a more than 1.5 folds change was considered differentially expressed. Pathway and network analyses were performed using Ingenuity Pathway Analysis (IPA) software. IPA computes a score for each network according to the fit of the set of supplied focus genes. These scores indicate the likelihood of focus genes belonging to a network versus those obtained by chance. A score > 2 indicates a < 99% confidence that a focus gene network was not generated by chance alone. The canonical pathways generated by IPA are the most significant for the uploaded data set. Fischer’s exact test with FDR option was used to calculate the significance of the canonical pathway.

For circRNA expression analysis, the reads were mapped to the genome using STAR [55]. DCC [56] was used to identify circRNA and to estimate the circRNA expression. TMM (trimmed mean of M-values) was used to normalize gene expression. Differentially expressed genes were identified using the edgeR program. miRanda [57] was used to predict miRNA targets of the circRNA. R was used to generate the figures.

### CircRNA verification by quantitative real-time polymerase chain reaction (qRT-PCR)

To validate the reliability of high-throughput RNA sequencing and to explore the expression of circRNAs during aging, the expression levels of circRNAs were examined by qRT-PCR. With reference to Memczak’s method [58], two sets of primers for each circRNA were designed using Primer Express software version 5.0 (Supplementary Table 2): an outward-facing set which was expected to amplify only the circRNA, and an opposite-directed set to amplify the linear form.

Total RNA was extracted (TRIzol® Reagent, Life technologies), digested using RNase R, and purified. cDNA was synthesized using a Geneseed^®^ II First Strand cDNA Synthesis Kit (Geneseed, USA). Outward-facing primers were designed to amplify the fragment across the junction from cDNA, then the fragment was sequenced by Sangon Biological Engineering Company (Shanghai China). QRT-PCR was performed using Geneseed^®^ qPCR SYBR^®^ Green Master Mix (Geneseed, USA), and PCR-specific amplification was conducted with an ABI 7500 (Applied Biosystems, USA). The expression of circRNAs was defined based on the threshold cycle (Ct), and relative expression levels were calculated via the 2^-ΔΔCt^ method. GAPDH served as an internal standard control with all reactions performed in triplicate.

### Cell cycle, apoptosis, proliferation, and autophagy evaluation

An astrocyte over expressing circNF1-419 was prepared. Its influence on cell cycle, apoptosis, and proliferation was evaluated as described [59], Wang K et al., 2016. Autophagy levels were measured by western blot and confirmed by transmission electron microscopy. Briefly, cells were fixed with 2.5% glutaraldehyde in 0.1 M sodium cacodylate buffer and stored at 4°C until embedding. The cells were post fixed with 1% OsO_4_ in 0.1 M cacodylate buffer (pH 7.2) containing 0.1% CaCl_2_ for 1 h at 4°C. After rinsing with cold distilled water, cells were dehydrated through a graded series of ethanol (30% – 100%). The samples were embedded in Embed-812 (EMS, 14120). After polymerization of the resin at 60°C for 36 h, serial sections were cut using an ultramicrotome (Leica) and mounted on formvar-coated slot grids (EMS, GA300-Cu). Sections were stained with 4% uranyl acetate and lead citrate, and examined with a Tecnai G2 F20 S-TWIN transmission electron microscope (FEI).

### Western blotting

Cells were seeded into 6-well culture plates at 5 × 10^6^ cells/well, and were washed twice with D-Hanks solution when the cells reached 80% confluence. The cells were harvested and lysed with protein lysis buffer and the protein concentration determined using a Coomassie Brilliant Blue G250 assay kit (Nanjing JianCheng Bioengineering Institute, China). Levels of PI3Kp85 (Protein, 60225-1-AP), PI3Kp100 (Protein, 60224-1-AP), AMPK (abcam, 80039), p53 (abcam, 66064), Erk1/2 (abcam, 17942), Atg13, ULK1 (abcam, 167139), Beclin-1 (Protein, 11306-1-AP), Atg14 (Protein, 19491-1-AP), Atg5 (Protein, 10458-1-AP), Atg12 (Protein, 1825-1-AP), LC3A (abcam, 128025), LC3B I, and LC3B II proteins were assessed by western blot with band intensity quantified using ImageJ software (NIH) as described previously [25]. Briefly, global brain tissue was dissected from treated mice (purchased from the Beijing HFK Bioscience Co., LTD [Certificate No: SCXK (Jing) 2014-0004]) and proteins extracted with radioimmunoprecipitation assay (RIPA) lysis buffer (Thermo Scientific^TM^ T-PER^TM^ Tissue Protein Extraction Reagent, 78510). The proteins were separated by sodium dodecyl sulfate-polyacrylamide gel electrophoresis and transferred onto polyvinylidene fluoride membranes. After blocking with 5% nonfat dry milk in Tris-buffered saline (20 mM Tris-HCl, 500 mM NaCl, pH 7.4) with 0.2% Tween-20 (Aladdin, T104863), the membranes were probed with antibodies overnight at 4°C, followed by incubation with a horseradish peroxidase-conjugated goat anti-mouse (Servicebio, G2211-1-A) or goat anti-rabbit (Servicebio, G2210-2-A) IgG secondary antibody (1:2000). The antibodies were as follows; anti-Abeita A4, -APOE, -BACE1, -p53 (abcam, 66064), -p16 (Affinity, AF0228), -p21, -p-Tau-396, -TNF-α (abcam, 9739), -p-Tau-202, obtained from Affinity as well as GAPDH (CST, 2118L) and β-Actin (CST, 4970S). Band intensity was quantified using ImageJ software (NIH).

The differentially expressed proteins were quantified using Wes™ and the Simple Western from ProteinSimple of RNA pull down samples [60].

### Histopathology and immunostaining

The brains of animals were dissected. A total of four brains from each group were fixed in 4% paraformaldehyde solution and prepared as paraffin sections. Sections were stained with hematoxylin-eosin (H&E), and immunostained for LC3A, Tau, p-Tau, Aβ A4, APOE, and BACE1 using paraffin-embedded 3 μm sections and a two-step peroxidase conjugated polymer technique (DAKO Envision kit, DAKO, Carpinteria, CA). Slides were observed by light microscopy (Chen et al., 2014; Zeng et al., 2013).

### RNA pull-down assay

Based on a previous study [59], interaction between specific proteins and circNF1-419 can be detected using a Biotin RNA probe. Briefly, based on the sequence of the circNF1-419 introns, a biotin-labeled specific pull down probe was designed and synthesized. The biotin-labeled RNA probe (1 μg) was denatured to form secondary structure, and 40 μl of magnetic beads were added to prepare a probe–magnetic bead complex. Brain tissues treated with an RNA interfering system (si*circNF1-419*-AAV) and an over-expressing *circNF1-419* system (ss*circNF1-419*-AAV) were collected and whole proteins were extracted for RNA pull-down. After interaction of the RNA-binding proteins with RNA, the samples were washed and the RNA binding protein complexes eluted. The samples were collected and 15 μl of each sample was subjected to liquid chromatography–mass spectrometry (LC-MS) and western blot analysis.

### RNA binding protein immunoprecipitation assay (RIP)

After circRNA pull down, the RNA binding protein (RBP) immunoprecipitation (RIP) assay was carried out [59]. Briefly, brain tissues were harvested with RIPA lysis buffer and sheared mechanically using a homogenizer. Biotin-labeled binding protein antibodies were added to cell extracts and incubated overnight at 4°C, followed by the addition of streptavidin-coated magnetic beads, and incubation for a further 4 h at 4°C. The magnetic beads were pelleted, washed and re-suspended in 1 mL Trizol. The isolated RNA was dissolved in 10 -20 μl of diethyl pyrocarbonate (DEPC) and circNF1-419 measured by qRT-PCR.

### Statistical analysis

Results from this study are presented as means ± SEM. Statistical analysis was performed using a two-tailed Student’s t test. A *p*-value < 0.05 was considered statistically significant.

### Ethics approval

The animal protocols used in this work were approved by the Institutional Animal Care and Use Committee of the Center of Laboratory Animals of the Guangdong Institute of Microbiology.

## Supplementary Material

Supplementary Figures

Supplementary Table 1

Supplementary Tables 2 and 3

Supplementary Table 4
